The article "Examination of bio convection with nanoparticles containing microorganisms under the influence of magnetism fields on vertical sheets by five-order Runge-Kutta method" was retracted in 2025. Reasons: unreliable results or conclusions; concerns about the authorship.

# Examination of bio convection with nanoparticles containing microorganisms under the influence of magnetism fields on vertical sheets by five-order Runge-Kutta method

**DOI:** 10.1016/j.heliyon.2023.e15982

**Published:** 2023-05-12

**Authors:** Reza Fathollahi, As'ad Alizadeh, Yaghub Safari, Hossein Nabi, Mahmoud Shamsborhan, Fariborz Taghinia

**Affiliations:** a Depatment of Engineering, Faculty of Khoy, Urmia University of Technology, Iran; b Department of Civil Engineering, College of Engineering, Cihan University-Erbil, Erbil, Iraq; c Department of Mechanical Engineering, Babol Noshirvani University of Technology, Babol, Iran; d Department of Mechanical Engineering, College of Engineering University of Zakho, Zakho, Iraq

**Keywords:** Bio convective fluid, Microorganisms, Nanofluid, Magnetic field, Vertical plate

## Abstract

In this paper, we analyzed vertical bio convection in nanofluids containing microorganisms. The novelty of this article is the numerical and analytical investigation of magnetic flow, radiation heat transfer, and viscous dissipation on bio convective fluid flow using the Five-order Runge-Kutta technique. Utilizing similitude parameters, determined ODE (ordinary differential equation) equations from partial differential equations for continuity, momentum, energy, and nanofluid concentration. Five-order Runge-Kutta was then used to solve the equations. The results show that it has a more significant influence on and then and. In addition, it exerts a force on neighboring particles, which causes them to shift from a hot zone to a great region. The density of microorganisms inside a part rises as it grows; when Le rises and *Ha* remains the same, x(ξ) falls, and When *Ha* rises, and Le remains the same, x(ξ) fall.

## Nomenclature

$\tilde{u},\tilde{v}$: =velocitycomponent
$\tilde{C}$: Nano fluid concentration (mg/cm3)
X,y,z: Coordinate directions
$\tilde{C}$*w*: Concentration on the sheet
$\tilde{N}$*w*: Free stream intensity
$\tilde{T}$*m*: Concentration on the sheet
$\tilde{x}$: Concentration of microorganisms
${\tilde{D}}_{T}$: Diffusion coefficients for thermophoretic
${\tilde{D}}_{B}$: Diffusion coefficients for Brownian
${\tilde{D}}_{m}=$: Diffusioncoefficientsformicroorganisms
$\alpha^{*}$: Stefan Boltzman constant
$k_{1}$: Roseland's average absorption
b: Constant of chemo taxis
*Wc*: = Rate of cell movement
$\tilde{\alpha }$: Thermal diffusivity
ρ: Density
ξ: Non-dimensional coordinate
ψ: Function
$\tilde{T}$: Temperature (c)
Pr: Prandtel parameter (dimensionless)
Le: The Lewis parameter (dimensionless)
Lb: bio-Convective (dimensionless)
M: magnetic interaction
Rd: radiation
Nb: Brownian motion
Yt: Thermal relaxation
Nt: Thermophoretic
*Pe*: Peclet number
Mb: Melting HT parameter
Nu_x_: Nusselt numeral
C_fx_: skin friction coefficient
Nx: Density number for motile microorganisms
Shr_x_: Sherwood number
t: Time component
$\tilde{u}$_e_: Free-fluid velocity
ρ: Density
B(x): Magnetism variable
σ: Stress component
$\lambda_{1}$: Dimensionless parameter
N: Rotating velocity

## 1 Introduction

In recent decades, studying nanoparticles has revealed a new objective for scientists. Nanofluids are, by convention, another sort of nanoparticle that binds this through conventional filter liquids (oils, water, gels, and polymers). Typically, these nanoparticles consist of metals, oxides, starchy polysaccharides, carbides, and non-metals and range in size from 1 to 100 nm.

Bio convection is a novel class of fluid mechanics and biology in which bio convection originates from macroscopic convective movements in a fluid caused by the addition of upwardly moving microorganisms (denser than the environment). Thus, self-propelled microorganisms loaded accumulate on the upper surface of the liquid and thus lead to varying density layering, directing to the emergence of bio-convection columns. Bio convection can be used in various applications such as B. Continuous refinement of biological polymer synthesis, eco-friendly applications, sustainable fuel cell technology, microbial-enhanced oil production, biosensors and biotechnology, and mathematical modeling in the pharmaceutical industry. Ali et al. [1] used Stephen's water-blowing and convective motions of thermal microorganisms to assess nano-sized metal pollutants to avoid fouling and degradation of the leading edges. The concentration of microorganisms and nanoparticles rose with melting, although the fluid's velocity and the temperature dropped as melting heat increased. On the upper horizontal surface of a rotating parabola, Makinde et al. [2] studied the affects of magnetism fields, nonlinear heat radiation, and homogeneous/heterogeneous quaternary autocatalysis on conductive alumina nanofluids (36 nm) harboring rotatotactic microorganisms. The velocity and density profiles of motile microorganisms are the Schmidt number reduction function. Ruchika et al. [3] analyze numerically the boundary layer flow of biotransformation and HT of electrically conductive nanofluids comprising nanoparticles and gyrotactic microorganisms on a sloping permeable sheet. Increasing the thermal slip and thermophores parameters decreases the HT rate. Makinde et al. [4] Investigate the combined effects of thermophoresis, thermal radiation, Brownian motion, variable viscosity, and magnetic fields on boundary layer flow, MT, and heat of conducting nanofluids on heated radially distorted convective surfaces. Rises in viscosity, radiation, convection, and nanofluid characteristics lead to a decrease in the rate of skin friction reduction as the magnetic field strength increases. The HT/MT rate and mobile microorganisms in the convective tensile flow of nanofluids made up of nanoparticles and gyrotactic microorganisms are investigated by Alsaedi et al. in their study published in Nature Communications [5]. The bigger the *Ha* and alpha, the less the velocity profile increases, and the more the concentration profile increases. The main subject of Shafiq et al. [6] is analyzing the heat and MT rate and moving microorganisms during the tangential hyperbolic material's hydrodynamic tangential convection (MHD). In the presence of both exponential surface nanoparticles, they conducted the investigation. The inclination angle and magnetic parameter are reduced functions of the velocity profile. Khan et al. [7] studied the mechanisms of unstable MT and HT in a hydrodynamic magnetic nanofluid (MHD) induced by a permeable tensile surface. The effects of Brownian motion and thermophoresis are combined in this scenario by the Buongiorno model. The varying parameters and MT effects for shear thinning and thickening fluids exacerbated the velocity, temperature, and dimensionless profiles. Raju et al. [8] present a numerical simulation investigating viscosity loss, temperature-dependent viscosity, and heat source/sink effect on unstable magnetohydrodynamic nanofluid (MHD) on a cone full of different alloy nanoparticles. The flow of a fully evolved mixture is evaluated in a porous media saturated with a nanofluid in the suspension of nanoparticles and microorganisms and led by its top moveable band wall. Hang et al. [9] investigated the mechanism of heat and MT caused by slip parameters, permeability, Brownian diffusion, thermophoresis, and bio-convection diffusion. Chakraborty et al. [10] examined the combined effects of convective boundary conditions and magnetic field on the natural convection of a nanofluid flow with an expanding plate containing gyro tactical microorganisms. As the thickness of the impulse boundary layer increases with M, the HT rate and flow velocity of the moving microorganism across the fluid medium decreases. It can also be explained that the velocity in the far field and the concentration of nanoparticles increased with M. Qayyum et al. [11] studied the rate of HT, concentration, and mobile microorganisms in the nanofluid radiation flow. By combining the effects of a magnetic field and buoyancy forces, natural convection is formed, stabilizing the idea of suspended nanoparticles of microorganisms. It is evident that with greater Brownian motion parameters, temperature and concentration react oppositely. Zaman et al. [12] investigate the bio convection Magnetohydrodynamic flow (MHD) of Williamson nanomaterials in the context of gyrotactic microorganisms. The density number increases through the physical displacement of the Schmidt number. A mathematical model is presented by Khan et al. [13] to investigate the flow of a water-based nanofluids natural convection boundary layer containing gyrotactic microorganisms on a short cone with surface convection boundary conditions. It was found that the densities of Sherwood number, motile microorganisms, skin friction, and Nusselt number increased along the surface. Nadeem et al. [14] focus on a viscous fluid's three-dimensional unstable bio-convective flow. An incompressible flow from a micro-polar nanofluid holds microorganisms next to an exponential magnetic field plane. The findings demonstrate that when the quantity of microorganisms rises, wall shear stress and Nusselt number drop. Tlili et al. [15] analyze the effect of bio-convective micropolar nanofluid flow consisting of gyrotactic microorganisms with thermal and soluble layering at the boundary surface. It turns out that the local density number worsens for Le, Pe, and bio convection. It is also observed that the velocity of the fluid decreases by increasing the bioconvective Rayleigh number. Naz et a [16]; investigate the entropy generated in the magnetohydrodynamic flow (MHD) of Williamson quasi-plastic nanofluid, including gyrotactic moving microorganisms on a tensile cylinder affected by an inclined magnetic field. The results show that the increased values of the Williamson fluid parameter reduce the velocity components for both the Newtonian and non-Newtonian states. The axial component of velocity increases with higher values of the thermal Grashof number, but the opposite behavior is observed for the condition of the temperature profile. Within the nearness of microorganisms and nanoparticles on surfaces, Hosseinzadeh et al. [17] examined Magnetohydrodynamic stream (MHD). As the Brownian movement increments from 0.1 to 0.9, the dimensionless temperature increments by 31.7%. In addition, by increasing the Schmidt number of bio-convection from 0.1 to 2, the characteristics of dimensionless microorganisms are reduced by more than four times. Alshomrani et al. [18] developed a mathematical model to visualize the non-Newtonian magnetic nanofluid cross-flow with MT rates of heat and activation energy, mobile microorganisms, and bioconvection on the wedge. It is discovered that the velocity decreases for the Rayleigh and bio-convection buoyancy ratio parameters while rising with the mixed convection parameter. Additionally, as activation energy parameter estimations are increased, so is the volumetric concentration of nanoparticles. The time-dependent three-dimensional thermal flow of a Maxwell nanofluid containing gyrotactic microorganisms is described by Ahmad et al. in Ref. [19]. Observations show that a decrease in both velocity components occurs due to the magnetic parameter. The velocity for the bio-convection Rayleigh number and the fixed buoyancy ratio in the horizontal direction tends to decrease. Aldabesh [20] examines the unstable flow of Williamson nanofluids containing gyrotactic microorganisms on a rotating cylinder. The concentration and distribution of microorganisms increase with the instability parameter. The mixed Pe, convection parameter, and Le of bio convection are associated with reducing microorganisms. Khan et al. [21] produced a two-way stream of Eyring-nanofluid Powell containing gyroscopic microorganisms by moving through a permeable plate subjected to thermal radiation and surface fascination. Suction brings down the temperature whereas quickening the HT. Additionally; the attraction velocity can be compensated by inducing a magnetic field in the flow field. By increasing thermophoretic and Brownian motion, the temperature distribution of Brownian motion grows more rapidly than that of thermophoretic motion and the nanoparticle volume fraction. Habibishandiz et al. [22] examined the convective heat transport of a mixed MHD nanofluid, including oxytactic microorganisms inside a vertical annular porous cylinder for the first time. It is concluded that the nearness of microorganisms leads to impeded HT, though expanded Hartmann numbers lead to made strides cruel Nusselt numbers. A Sutterby nanofluid with connected attractive field and a convective boundary component known as two coaxial pivoting footing circles were proposed by Waqas et al. Inspected [23]. The flow velocity is accelerated directly by the mixed convection parameter but is delayed by the magnetic field parameter and the bio convection Rayleigh number. Temperature ratio, biot number, thermophoresis, and thermal conductivity factors all increase fluid temperature. On straight extension plates in which rotatative microorganisms reside, Sankad et al. [24] the aim is to investigate the combined effects of magnetic and convective boundary conditions on bio convection and nanoparticle concentrations in Kasson fluids. An increase in fluid temperature occurs due to ascending values of Brownian motion, thermophores, and thermal Rd s. Prandtl number and suction parameter reduce fluid temperature. The magnetic field parameter raises the concentration of nanoparticles in the current while the Le and suction parameter decrease. Famakinwa et al. [25] conducted a numerical analysis of changes in viscosity, thermal radiation, and Arrhenius reaction on the flow of an electrically conductive nanofluid via a heated convective surface. It was discovered that a rise in the parameter of viscosity changes enhances the velocity gradient and velocity of HT but reduces the MT rate and density of mobile microorganisms at various values of Rd and Kr. In addition, increasing the rate of the chemical reaction decreases the concentration distribution, but the concentration distribution grows with increasing heat radiation. Habibishandiz et al. [26] investigate MHD nanofluid, including oxytocic microorganisms, inside a porous cylinder. Increasing the Hartman number considerably improves heat transmission in the presence of microorganisms, as demonstrated by the study's findings. According to Naganthran et al. [27], boundary layer flow, heat, mass, and the transfer of live microorganisms from a porous tensile surface in an expanding nanofluid are all affected by magnetohydrodynamic (MHD) and chemical reactions. Different types of slips on the tensile sheet's surface affect the mechanisms adjacent to the boundary layer. The velocity of the fluid in a tensile sheet is decreased by increasing the velocity slip parameter for dilatant and Newtonian nanofluids. For dilatant and Newtonian nanofluids, a rise in the mass field extremely near the plane is seen as the mass slip parameters are increased. The nanoparticle volume fraction on the tensile sheet decreases when the chemical reaction parameter is increased. The more considerable magnetic force increases the local Sherwood number and skin friction. Elayarani et al. [28] present mathematical and adaptive models of the fuzzy neural inference system (ANFIS) for the unstable biodegradation flow of Carreau nanofluids, which presents the gyrotactic microorganisms on a narrow tensile plate with the presence of a magnetic field and multiple thermal radiation conditions. The coefficient of friction decreases with increasing Weisenberg number and velocity slip parameter. Heat transport is enhanced by raising the levels of thermal slip and Brownian motion. MT rises due to elevated thermophoresis and concentration slip parameters under the control of the process's Le. Waqas et al. [29] studied the rotational flow of the electrically conductive Oldroyd-B MHD fluid through an extracorporeal porous medium across a tensile/shrinking surface within the range of bio-convection effects. As the Deborah number, Biot number, buoyancy ratio parameters, rotation, porosity, magnetic field intensity, and diffusion of thermophores rise, it has been demonstrated that the fluid's temperature characteristics also increase. Hasibi et al. [30].'s analysis of the second-class Casson fluid convection in a microchannel influenced by an induced magnetic field and an exponential heat source. Kahn et al. [31] investigate an Oldroyd-B transient two-dimensional radiation nanofluid flow. The flow field is exposed to an exponentially elastic surface that is heated conventionally. It is demonstrated that the fluid velocity is decreased for greater values of the relaxation parameter while its behavior rises for larger values of the delay parameter. Additionally, greater values of the relaxation parameter match the maximum mass and rate of HT, while lower values match the delay parameter. Non-Newtonian blood liquid flow with nanoparticles interior a porous-walled pipe was explored by Hosseinzadeh et al. [32] within the nearness of a magnetism field. Hussain et al. [33] discussed the self-traction motion of gyrotactic swimmer microorganisms during the generalized slip of the MHD nanofluid next to a tensile cylinder. Higher value of the ebb and flow parameter and the Richardson number conclusion in an increment in velocity. In contrast, it is decreased at certain places in the amplitude by the bio convection Rayleigh number, the buoyancy ratio, the magnetic field, and the slip parameters [[34], [35], [36], [37], [38], [39], [40], [41]]. Biswas and his colleagues conducted many researches and studies about the effects of magnetic current created on systems and porous plates under the influence of fluid flows and bio-nanofluids. According to one of the results obtained from their research, the general patterns of fluid flow, temperature, and distribution of oxygen and microorganisms were markedly affected by increasing magnetic field strength [[42], [43], [44], [45]].

In this research, we analyzed the flow of bioconvective fluids containing microorganisms and nanoparticles. The governing equations include the effects of the magnetic field, thermal radiation, and viscous dissipation. Five-order Runge-Kutta was then utilized to solve the equations. The influence of magnetic field on various velocity profiles, temperature, nanofluid concentration, microbe concentration, Nusselt number, and skin friction has been studied. **An innovation in this work is the numerical and analytical study of magnetic flux, radiative heat transfer, and viscous dissipation for bio convective fluid flow using the fifth-order Runge-Kutta method, which is also the first to use this method to demonstrate vertical bioconvective microbes. In this work, mixtures containing ethylene glycol water and Fe3O4 were investigated.**

## 2 Scientific definition of the issue

Here, an incompressible and unstable viscous nanofluid is assumed to flow through a semi-infinite rigid static plate, causing leading edge attachment/erosion. Gyrotactic microorganisms have a role in potentially precipitating micron-sized metal compounds by stemming (blocking) this process (Table 1). Additionally, melting heat's consequences are mentioned. (See Refs. [46,47]). The magnetic field used across acute angle ***β***, and it is supposed to be a distance function from the origin indicated as (*x*) = *Bo*∕(***ν****t*cos***α*** + (*U****ν****x* $\tilde{\infty }$)sin***α***)1∕2, here *Bo* ≠ 0. In the current investigation, the free-stream velocity is denoted by the symbol $\tilde{U}$ ∞. Additionally, it was taken into account that the free stream intensity is $\tilde{N}$ ∞, $\tilde{C}$ ∞, and temperature T, respectively, and that the concentration and temperature on the sheet are $\tilde{C}$ *w*, $\tilde{N}$ *w*, and $\tilde{T}$ *m*, respectively. Using the coordinate system (x, y) is also appropriate, where x is parallel to the sheet and y is vertical (see Fig. 1). The model's governing equations for the present modeled issue are as follows [2,46,47]:

(1) $$\frac{\partial \tilde{v}}{\partial y}+\frac{\partial \tilde{u}}{\partial x}=0$$

(2) $$\frac{\partial \tilde{u}}{\partial t}+\tilde{v}\frac{\partial \tilde{u}}{\partial y}+\tilde{u}\frac{\partial \tilde{u}}{\partial x}={\tilde{u}}_{e}\frac{\partial {\tilde{u}}_{e}}{\partial x}+\frac{\partial {\tilde{u}}_{e}}{\partial t}+v\frac{\partial^{2}\tilde{u}}{{\partial y}^{2}}-\frac{\sigma B\left(x\right)}{\rho }\sin^{2}\;\beta \left(\tilde{u}-{\tilde{U}}_{\infty }\right)$$

(3) $$\frac{\partial \tilde{T}}{\partial t}+\tilde{v}\frac{\partial \tilde{T}}{\partial y}+\tilde{u}\frac{\partial \tilde{T}}{\partial x}+\lambda_{1}T_{\lambda }=\tilde{\alpha }\frac{\partial^{2}\tilde{T}}{{\partial y}^{2}}-\frac{\partial q_{r}}{\partial y}+\left({\tilde{D}}_{B}\frac{\partial \tilde{T}}{\partial y}\frac{\partial \tilde{C}}{\partial y}+\frac{{\tilde{D}}_{T}}{{\tilde{T}}_{\infty }}{\left(\frac{\partial \tilde{T}}{\partial y}\right)}^{2}\right)$$

(4) $$\frac{\partial \tilde{C}}{\partial t}+\tilde{v}\frac{\partial \tilde{C}}{\partial y}+\tilde{u}\frac{\partial \tilde{C}}{\partial x}+\lambda_{1}T_{\lambda }={\tilde{D}}_{B}\frac{\partial^{2}\tilde{C}}{{\partial y}^{2}}+\frac{{\tilde{D}}_{T}}{{\tilde{T}}_{\infty }}\frac{\partial^{2}\tilde{T}}{{\partial y}^{2}}$$

(5) $$\frac{\partial \tilde{N}}{\partial t}+\tilde{v}\frac{\partial \tilde{N}}{\partial y}+\tilde{u}\frac{\partial \tilde{N}}{\partial x}+\left[\frac{\partial }{\partial y}\left(\tilde{N}\frac{\partial \tilde{C}}{\partial y}\right)\right]\frac{\left(b\right)Wc}{\left({\tilde{C}}_{\omega }-{\tilde{C}}_{\infty }\right)}=D_{m}\frac{\partial^{2}\tilde{N}}{{\partial y}^{2}}$$

(6) $$T_{\lambda }=\tilde{u}\frac{\partial \tilde{u}}{\partial x}\frac{\partial \tilde{T}}{\partial x}+\tilde{u}\frac{\partial \tilde{v}}{\partial x}\frac{\partial \tilde{T}}{\partial y}+\tilde{v}\frac{\partial \tilde{v}}{\partial y}\frac{\partial \tilde{T}}{\partial y}+2\tilde{u}\tilde{v}\frac{\partial^{2}\tilde{T}}{\partial y\partial x}+\tilde{u^{2}}\frac{\partial^{2}\tilde{T}}{{\partial x}^{2}}+\tilde{v^{2}}\frac{\partial^{2}\tilde{T}}{{\partial y}^{2}}$$

(7) $$\tilde{u}=0,\tilde{v}=0,\tilde{T}=T_{w},\tilde{C}={\tilde{C}}_{w},\tilde{N}={\tilde{N}}_{w},aty=0$$

(8) $$\tilde{u}\to {\tilde{U}}_{\infty },\tilde{T}\to {\tilde{T}}_{\infty },\tilde{C}\to {\tilde{C}}_{\infty },\tilde{C}\to {\tilde{C}}_{\infty },aty\to \infty$$

**Table 1:** Thermo-physical properties of base fluid and nanoparticles.

Physicalproperties	Ethylene glycol-Water	Water	Fe_3_O_4_
$\rho \;\left(\frac{kg}{m^{3}}\right)$	1063.8	997.1	4250
$c_{p}\;\left(\frac{J}{kg.^{\circ }K}\right)$	3630	4179	686.2
$k\;\left(\frac{W}{m.^{\circ }K}\right)$	0.387	0.613	8.9538

**Fig. 1:** Geometry of the problem.

If 1 = 0, Equation (3) transforms into the Fourier equation. In addition, ($\tilde{u}$) and ($\tilde{v}$) denote the components of velocity along the x and y dimensions, respectively, and are represented by temperature T, the volume gradient of nanoparticles C, t is the time component, u $\tilde{e}$ is the free-fluid velocity, ρ is the density, B(x) is the Magnetism variable, σ is the stress component, $\lambda_{1}$ is the dimensionless parameter, N is the rotating velocity, and the concentration of microorganisms $\tilde{\chi }$. In addition, ${\tilde{D}}_{T}$, ${\tilde{D}}_{B}$, and ${\tilde{D}}_{m}$ collectively represent the diffusion coefficients for thermophoretic, Brownian, and microorganisms. In addition, q_r_ is given as $q_{r}=\frac{4}{3}\frac{\alpha^{*}}{K_{1}}\frac{\partial {\tilde{T}}^{4}}{{\partial y}^{2}}$, where $\alpha^{*}$ is the Stefan Boltzman constant and K_1_ is Roseland's average absorption, b is the constant of chemotaxis, and W_c_ is the rate of cell movement. Additionally, $\tilde{\alpha }$ represent thermal diffusivity. Initial and boundary conditions related with the issue are as follows [2,46]:

Proposing the aforementioned similarity vectors as follows: ([29,31,32]):

$$\Psi ={\tilde{U}}_{\infty }f\left(\xi \right)\sqrt{\left(vt\right)\cos\;\alpha +\left(\frac{vx}{{\tilde{U}}_{\infty }}\right)\sin\;\alpha }\text{,}$$

$$\theta \left(\xi \right)=\frac{\left\{\tilde{T}-{\tilde{T}}_{\infty }\right\}}{\left\{{\tilde{T}}_{w}-{\tilde{T}}_{\infty }\right\}}\text{,}$$

(9) $$\varphi \left(\xi \right)=\frac{\left\{\tilde{C}-{\tilde{C}}_{\infty }\right\}}{\left\{C_{w}-{\tilde{C}}_{\infty }\right\}}\text{,}$$

$$\chi \left(\xi \right)=\frac{\tilde{N}}{{\tilde{N}}_{w}}\text{,}$$

$$\xi =\frac{y}{\sqrt{\cos\;\alpha \left(tv\right)+\sin\;\alpha \left(\frac{vx}{{\tilde{U}}_{\infty }}\right)}}\text{,}$$

The non-dimensional coordinate is ξ, α is fixed and ψ is a function of $\tilde{u}=\frac{\partial \psi }{\partial y}$ and $\tilde{v}=\frac{\partial \psi }{\partial x}$ that fulfills the equation of the non-dimensional coordinate (1). The nonlinear ODEs discussed below may be derived from equations (2)–(8) using equation (9) [[2], [3], [4], [5], [6], [7], [8], [9], [10], [11], [12], [13], [14], [15], [16], [17], [18], [19], [20], [21], [22], [23], [24], [25], [26], [27], [28], [29], [30], [31], [32], [33], [46], [47], [48]].

(10) $$f^{\prime \prime \prime }+\frac{1}{2}\sin\;\alpha ff^{\prime \prime }+\frac{1}{2}\cos\;\alpha \xi f^{\prime \prime }+M\;\sin^{2}\;\beta -M\;\sin^{2}\;\beta f^{\prime }=0$$

(11) $${\left(1+Rd\right)\theta }^{\prime \prime }+\frac{1}{2}\mathrm{Pr}\left(\xi \theta^{\prime }\;\cos\;\alpha +f\theta^{\prime }\;\sin\;\alpha \right)+Nb\theta^{\prime }\varphi^{\prime }+Nt{\theta^{\prime }}^{2}+\frac{\mathrm{Pr}}{2}\gamma_{T}\left(\theta_{rT}\right)=0$$

(12) $$\varphi^{\prime \prime }+\frac{1}{2}PrLe\left(\xi \varphi^{\prime }\;\cos\;\alpha +f\varphi^{\prime }\;\sin\;\alpha \right)+\frac{Nt}{Nb}\theta^{\prime \prime }=0$$

(13) $$\chi^{\prime \prime }+\left\{\frac{\xi \chi^{\prime }}{2}\cos\;\alpha +\frac{f\chi^{\prime }}{2}\sin\;\alpha \right\}\left(LbPr\right)-Pe\left(\chi \varphi^{\prime \prime }+\chi '\varphi '\right)=0$$

$$f^{\prime }\left[\xi \right]=0,M_{b}\theta^{\prime }\left(\xi \right)+\frac{\mathrm{Pr}}{2}\sin\;\alpha f\left(\xi \right)=0,\varphi \left[\xi \right]\to 1,\theta \left[\xi \right]\to 1,\chi \left[\xi \right]=1at\;\xi =0$$

(14) $$f^{\prime }\left[\xi \right]\to 1,\varphi \left[\xi \right]\to 0,\theta \left[\xi \right]\to 0,\chi \left[\xi \right]\to 0at\;\xi \to \infty$$

where $\theta_{\gamma T}=\left(3\;\sin\;aff^{\prime }\theta^{\prime }+\xi \;\sin\;af\theta^{\prime \prime }\right)$ appears in equation (10), (11), (12), (13), (14), the developing parameters are designated as [[2], [3], [4], [5], [6], [7], [8], [9], [10], [11], [12], [13], [14], [15], [16], [17], [18], [19], [20], [21], [22], [23], [24], [25], [26], [27], [28], [29], [30], [31], [32], [33], [46], [47], [48]]:

$$\frac{v}{\tilde{\alpha }}=\mathrm{Pr},\frac{\tilde{\alpha }}{{\tilde{D}}_{B}}=Le,\tilde{\alpha }{\left\{{\tilde{D}}_{m}\right\}}^{-1}=Lb,Rd=16\sigma^{*}\frac{{\tilde{T}}_{\infty }^{3}}{3k^{*}K},M=\frac{\sigma B_{0}^{2}}{\rho },\tau {\tilde{D}}_{B}{\tilde{\alpha }}^{-1}\left({\tilde{C}}_{w}-{\tilde{C}}_{\infty }\right)=Nb,\tau {\tilde{D}}_{T}{\left(\tilde{\alpha }{\tilde{T}}_{\infty }\right)}^{-1}\left({\tilde{T}}_{w}-{\tilde{T}}_{\infty }\right)=Nt,\gamma_{T}=\lambda_{1}{\tilde{U}}_{\infty },Pe=\frac{bWc}{Dm},Mb=\frac{Cp\left({\tilde{T}}_{w}-{\tilde{T}}_{\infty }\right)}{\lambda_{1}+Cs\left({\tilde{T}}_{m}-{\tilde{T}}_{0}\right)}$$

The Lewis, Prandtl, and bio-Convective Le are represented as Le, Pr, and Lb, whereas the magnetic interaction, radiation, Brownian motion, thermal relaxation, and Nt s are represented as M, Rd, Nb, $\gamma_{T}$, N t. Also expressed as *Pe* and Mb are the bio-convection Péclet number and melting HT parameter, respectively. The local Nusselt number (Nu_x_), local expressions of skin friction coefficient (Cf_x_), density number for motile microorganisms (N_x_), and Sherwood number (Shr_x_) have been categorized as follows [[2], [3], [4], [5], [6], [7], [8], [9], [10], [11], [12], [13], [14], [15], [16], [17], [18], [19], [20], [21], [22], [23], [24], [25], [26], [27], [28], [29], [30], [31], [32], [33], [46], [47], [48]].:

$$Cf_{x}=\frac{\mu }{\rho {\tilde{U}}_{\infty }}{\left[\frac{\partial \tilde{u}}{\partial y}\right]}_{y=0},{Nu}_{x}=\frac{-x}{\left({\tilde{T}}_{w}-{\tilde{T}}_{\infty }\right)}{\left[\frac{\partial \tilde{T}}{\partial y}\right]}_{y=0}+q_{r}\text{,}$$

(15) $${Shr}_{x}=\frac{-x}{\left({\tilde{C}}_{w}-{\tilde{C}}_{\infty }\right)}{\left[\frac{\partial \tilde{C}}{\partial y}\right]}_{y=0},N_{x}=\frac{-x}{\left({\tilde{N}}_{w}-{\tilde{N}}_{\infty }\right)}{\left[\frac{\partial \tilde{N}}{\partial y}\right]}_{y=0}$$

It is obtained using the transformation vectors equation (8) as [[2], [3], [4], [5], [6], [7], [8], [9], [10], [11], [12], [13], [14], [15], [16], [17], [18], [19], [20], [21], [22], [23], [24], [25], [26], [27], [28], [29], [30], [31], [32], [33], [46], [47], [48]].:

(16) $$Cf_{x}{{Re}_{x}}^{\frac{1}{2}}{\left[\sin\;a+\tau \;\cos\;a\right]}^{\frac{1}{2}}=f^{\prime \prime }\left(0\right)$$

$${Nu}_{x}{{Re}_{x}}^{\frac{-1}{2}}{\left[\sin\;a+\tau \;\cos\;a\right]}^{\frac{1}{2}}=-\left(1+Rd\right)\theta^{\prime }\left(0\right)$$

$${Shr}_{x}{{Re}_{x}}^{\frac{-1}{2}}{\left[\sin\;a+\tau \;\cos\;a\right]}^{\frac{1}{2}}=-\varphi^{\prime }\left(0\right)$$

$$N_{x}{{Re}_{x}}^{\frac{-1}{2}}{\left[\sin\;a+\tau \;\cos\;a\right]}^{\frac{1}{2}}=-x^{\prime }\left(0\right)$$

where τ is a nondimensional time parameter and ${Re}_{x}=\frac{{\tilde{u}}_{\infty }x}{v}$ is the Reynolds number.

## 3 Numerical method

The**6-level order 5** Runge-Kutta method requires finding a matrix **A** whose coefficients must satisfy a system of nonlinear **polynomials.** Butcher found a **five-parameter** solution family that exhibits different **properties** depending on whether **b2** = 0 or b2, **0.** The Runge-Kutta calculation estimates the anticipated rates at various focuses within the time interval from t to **t** + **h. So if** the **rate** (differential **equation) explicitly depends** on **t,** we also need to know the value of t at those points **in** the time **interval**. An explicit Runge-Kutta method is never A-stable since the stability function of the exact Runge-Kutta method is polynomial. It is, therefore, interesting to examine the polynomial quotients of particular degrees that best approximate the exponential function. By adding boundary conditions and converting the nonlinear differential equations to first-order linear equations, we solve them using the fifth-order Runge-Kutta, Verberg method (24).

(17) $$\begin{array}{l} {\left(f,f^{\prime },f^{\prime \prime },f^{\prime \prime \prime }.g,g^{\prime },\theta ,\theta^{\prime },p\right)}^{T}=\\ {\left(y_{1},y_{1}^{\prime }=y_{2},y_{2}^{\prime }=y_{3},y_{3}^{\prime }=y_{4},y_{5},y_{5}^{\prime }=y_{6},y_{7},y_{7}^{\prime }=y_{8},y_{9}\right)}^{T}\text{.} \end{array}$$

The Runge-Kutta Fehlberg fifth order uses equation (17) for differential equation terms [[2], [3], [4], [5], [6], [7], [8], [9], [10], [11], [12], [13], [14], [15], [16], [17], [18], [19], [20], [21], [22], [23], [24], [25], [26], [27], [28], [29], [30], [31], [32], [33], [46], [47], [48]].

(18) $$\left(\begin{array}{l} y_{1}^{\prime }\\ y_{2}^{\prime }\\ y_{3}^{\prime }\\ y_{4}^{\prime }\\ y_{5}^{\prime }\\ y_{6}^{\prime }\\ y_{7}^{\prime }\\ y_{8}^{\prime }\\ y_{9}^{\prime } \end{array}\right)=\left(\begin{array}{l} y_{2}\\ y_{3}\\ y_{4}\\ {\left(1-\varphi \right)}^{2.5}\left(1-\varphi +\frac{\rho_{s}}{\rho_{f}}\varphi \right)\left[Re\left(2y_{1}y_{3}+2y_{5}y_{6}-\frac{M}{1-\varphi +\frac{\rho_{s}}{\rho_{f}}\varphi }y_{3}\right)\right]\\ y_{6}\\ \frac{1}{{\left(1-\varphi \right)}^{2.5}\left(1-\varphi +\frac{\rho_{s}}{\rho_{f}}\varphi \right)}g^{\prime \prime }+Re\left(2fg^{\prime }-2f^{\prime }g-\frac{M}{1-\varphi +\frac{\rho_{s}}{\rho_{f}}\varphi }g\right)\\ y_{8}\\ \mathrm{Pr}\left(\frac{k_{f}}{k_{nf}}+\frac{1}{k_{nf}}\right)\left[2Re\left(1-\varphi +\frac{{\left(\rho c_{p}\right)}_{s}}{{\left(\rho c_{p}\right)}_{f}}\varphi \right)y_{1}y_{8}+ReMEc\left({y_{2}}^{2}+{y_{5}}^{2}\right)\right] \end{array}\right)$$

(19) $$\left\{ \begin{array}{l} y_{1}\left(0\right)=W_{s},y_{2}\left(0\right)=A_{1},y_{3}\left(0\right)=z_{1},y_{4}\left(0\right)=z_{2},y_{5}\left(0\right)=1,y_{6}\left(0\right)=z_{3},y_{7}\left(0\right)=1\text{,}\\ y_{8}\left(0\right)=z_{4},y_{9}\left(0\right)=0\text{.} \end{array}\right.$$

The projected outcomes of this numerical method are almost entirely consistent with the scientific literature (see Table 2 and Fig. 2).

**Table 2:** Values of $F^{\prime }\left(0\right)$ in comparison with other researches according to α.

α	Current Results	[33]	[48]	[46]	[47]	[1]
0	0.564193162	0.564191	0.5642	0.564189	0.56418	0.56419
π/24	0.575016139	0.575018	0.575	0.575016	0.57501	0.575019
π/12	0.580728841	0.580731	0.5807	0.580728	0.58072	0.580726
π/6	0.577001466	0.577004	0.577	0.577001	0.577	0.577002
π/4	0.552874465	0.552877	0.5529	0.552875	0.55287	0.552876
π/3	0.507217839	0.50722	0.5072	0.507218	0.50721	0.507221
5π/12	0.436863707	0.436866	0.4369	0.436864	0.43686	0.436867
11π/24	0.389998689	0.39	0.39	0.389999	0.38999	0.390002
π/2	0.332057337	0.332059	0.3321	0.332057	0.33205	0.332057

**Fig. 2:** Comparison of present work with Hussain work [33] for $F^{\prime }\left(\varepsilon \right)$.

## 4 Comes about and converse

Fig. 3(a) and b depicts the exact influence of *Ha* on $F^{\prime }\left(\xi \right)$ with varying α and β values. The data in Figure indicate that with $\alpha =\frac{\pi }{4}$, the boundary layer domain's velocity decrease, and it thickens more than with $\alpha =\frac{\pi }{2}$. When α grows, and *Ha* remains the same, $F^{\prime }\left(\xi \right)$ decrease, and when *Ha* grows, and α remains the same, $F^{\prime }\left(\xi \right)$ increase. When β grows, and *Ha* remains the same, $F^{\prime }\left(\xi \right)$ increase generally. The change trends for the two BB values are congruent in some *Ha* values. With the increase of the Hartmann number, the velocity boundary layer will increase, and the velocity gradient will expand at different points of the plane.

**Fig. 3:** Effects of Hartman number on velocity with varying αinfig(a) and βinfig(b).

Fig. 4 depicts the exact influence of *Ha* on θ(ξ) with varying α, Nb, Nt and Rd values. The data in Fig. 4(a) indicate that when α grows, and *Ha* remains the same, θ(ξ) decrease and when *Ha* grows, and α remains the same, θ(ξ) increase. So, $F^{\prime }\left(\xi \right)$ is evidently most affected by *Ha* and α. Fig. 4(b) shows that *Ha* has a monotonically decreasing value relative to Nb, as seen by the schematic layout of these values. The melting process removes the achievement of heat fluxion and the volume fraction flux of the nanoparticles. Consequently, the growth of Nb in the constant *Ha* causes θ(ξ) decreases slightly. With unchanged Nb, an increase in *Ha* causes a slight rise in physically; Nt exerts a force on neighboring particles, which causes them to shift from a hot zone to an incredible region. As demonstrated in Fig. 4(c), the temperature increases with a slight increase in the Nt. Fig. 4(d) shows that an increase in the Rd has an ascending influence, as seen by the graphical representations of these data. Relatively, with the increase of the Hartmann number in different ranges from eta, the temperature values decrease insignificantly, and the thickness of the thermal boundary layer decreases. Also, around the wall, the temperature reaches the lowest degree.

**Fig. 4:** Effects of Hartman number on temprtature with varying stephabboltzman, Brownianmotrion, thermophoretic and Radiation.

Fig. 5 depicts the exact influence of *Ha* on φ(ξ) with varying α, , Nb, Nt and Rd values. Fig. 5(a) shows that when α grows, and *Ha* remains the same, φ(ξ) increase, and when *Ha* grows, and α remains the same, φ(ξ) decrease. Fig. 5(b) shows that when β grows, and *Ha* remains the same, φ(ξ) decrease. In the same way, When *Ha* grows, and β remains the same, φ(ξ) decrease. Fig. 5(c) shows that a growth of Nb in the constant *Ha* causes φ(ξ) to increase, and with unchanged Nb, an increase in *Ha* causes a drop in φ(ξ). Fig. 5(d) shows that with a slight increase in the Nt, the φ(ξ) decreases. In a physical sense, Nt exerts a force on nearby particles, causing them to relocate from a heated zone to a cold zone.

**Fig. 5:** Effects of Hartman number on φ(ξ) with varying stephabboltzman, Brownianmotrion, thermophoretic and Radiation.

Fig. 6 depicts the exact influence of *Ha* on x(ξ) with varying α, , Nb, Nt,Pe, and Le values. Fig. 6(a) shows that when α grows, and *Ha* remains the same, x(ξ) increase and When *Ha* grows, and α remains the same, x(ξ) decrease. Fig. 6(b) shows that when β grows, and *Ha* remains the same, x(ξ) decrease. In the same way, When *Ha* grows, and β remains the same, x(ξ) decrease. *Ha* has a monotonically decreasing value relative to Nb, as seen by the schematic layout of these values. The melting process removes the achievement of heat fluxion and the volume fraction flux of the nanoparticles. Fig. 6(c) shows that the growth of Nb in the constant *Ha* causes x(ξ) to increase and with unchanged Nb, an increase in *Ha* causes a drop in x(ξ). As demonstrated in Fig. 6(d) the density of microorganisms inside a region rises as Nt grows. As demonstrated in Fig. 6(e–f), when Pe and Le grows, and *Ha* remains the same, x(ξ) decreases, and When *Ha* grows, and Pe and Le remains the same, x(ξ) decreases. According to Fig. 6, with the increase of the Hartmann number, the amount of concentration of nanofluids around the plate decreases. As the distance from the end to the beginning of the page decreases, the drop in concentration is noticeable, and the viscosity decreases.

**Fig. 6:** Effects of Hartman number on x(ξ) with varying stephabboltzman, Brownianmotrion, thermophoretic and Radiation,Pecletnumber and TheLewis Parameter.

Fig. 7 depicts the exact influence of *Ha* on Cf,Nu,Sh,Nx with varying β,Rd, Nt and Pe values. Fig. 7(a) shows that when β grows, and *Ha* remains the same, Cf increases. In the same way, When *Ha* grows, and β remains the same, x(ξ) increases. Fig. 7(b) shows that an increase in the Rd has an ascending influence on Nu, as seen by the graphical representations of these data. Fig. 7(c) shows that when Nt grows, and *Ha* remains the same, Sh decreases. In the same way, When *Ha* grows, and Nt remains the same, Sh increases. As demonstrated in Fig. 7(d), when Pe grows, and *Ha* remains the same, Nx increases, and When *Ha* grows, and Pe remains the same, Nx increases. All relevant calculations and simplifications implemented in this step are shown in the uncertainty analysis diagram in Fig. 8. According to the fluctuating temperature diagram obtained from the two methods (Fig. 9), the temperature parameter changes have been repeated alternately along the screen for a short interval of ξ. The accuracy of the solution is for minimal distances between the plates, and the thermal fluctuations have been obtained with macroscopic accuracy. The temperature values around the thermal boundary layer of the plate wall have molecular movements with high heat transfer, which increases the velocity gradient of the nanoparticle spread around the wall.

**Fig. 7:** Effects of Hartman number on skinfrictioncoefficient,Nusseltnumber,Sherwoodnumber,Densitynumberformotilemicroorganisms with varying β,radiation,thermophoretic and pecklet number.

**Fig. 8:** The Uncertainly Analysis chart.

**Fig. 9:** Oscillatory graph of the problem in a certain interval of the thermal boundary layer around the wall temperature for heat transfer by comparison between FEM and ADM.

## 5 Conclusion

In this paper, we analyzed vertical bio convection in nanofluids containing microorganisms. The novelty of this article is the numerical and analytical investigation of magnetic flow, radiation heat transfer, and viscous dissipation on bio convective fluid flow using the Five-order Runge-Kutta technique. Utilizing similitude parameters, determined ODE equations from partial differential equations for continuity, momentum, energy, and nanofluid concentration. Five-order Runge-Kutta was then used to solve the equations. The results show that, Re has a more significant influence on Cf and Nu than M and φ. In addition, Nt exerts a force on neighboring particles, which causes them to shift from a hot zone to a cool region, and the density of microorganisms inside a region rises as Nt grows.

• When α rises, and *Ha* remains the same, $F^{\prime }\left(\xi \right)$ and θ(ξ) fall, during x(ξ) and φ(ξ) grow.
• Nb alterations have a more significant impact on θ(ξ), φ(ξ) and x(ξ) than *Ha* changes.
• When Le rises, and *Ha* remains the same, x(ξ) fall, and When *Ha* rises, and Le remains the same, x(ξ) fall.
• The density of microorganisms inside a region increases as Nt rises.
• The grow in the radiation parameter (Rd) had a descending influence on θ(ξ).
• Re Has a greater influence on Nu and Cf than M and φ.

## Author contribution statement

Reza Fathollahi: Contributed analysis tools or data; Wrote the paper.

As'ad Alizadeh, Mahmoud Shamsborhan: Conceived and designed the analysis.

Yaghub Safari: Analyzed and interpreted the data.

Hossein Nabi: Analyzed and interpreted the data; Wrote the paper.

Fariborz Taghinia: Contributed analysis tools or data.

## Data availability statement

Data included in article/supp. material/referenced in article.

## Declaration of competing interest

The authors declare that they have no known competing financial interests or personal relationships that could have appeared to influence the work reported in this paper.
